# Implications of Ezetimibe in Combination with Low- to Moderate-Intensity Atorvastatin Adjuvant Aspirin Therapy for Cerebrovascular Disease

This article has been retracted.

**DOI:** 10.1155/2022/3369226

**Published:** 2022-07-18

**Authors:** Lijie Wang, Xiaoqin Tang

**Affiliations:** The People's Hospital of Suzhou New District, Department of Neurology, China

## Abstract

**Objective:**

To analyze the significance of ezetimibe in combination with low- to moderate-intensity atorvastatin adjuvant aspirin therapy for cerebrovascular disease.

**Methods:**

110 patients with cerebrovascular disease treated in our hospital from June 2020 to June 2021 were selected and divided into 55 patients in the control group and 55 patients in the study group according to the lottery method. After a comprehensive examination, patients in the two groups should be given aspirin for treatment; the control group was treated with conventional dose of atorvastatin on top of the above, and the study group was given ezetimibe and medium-low-dose atorvastatin on top of aspirin treatment, activities of daily living (ADL) score, carotid artery intima-media thickness, lipid level, coagulation level, clinical effect, and adverse rate of the two groups which were tested and compared.

**Results:**

After treatment, ADL score, high-density leptin cholesterol (HDL-C), and ATIII levels increased, while carotid artery media thickness, triglyceride (TG), total cholesterol (TC), low-density leptin cholesterol (LDL-C), DD, PC, and hs-CRP levels decreased (*P* < 0.05). After treatment, ADL score, HDL-C, and ATIII levels were higher in the study group. The levels of carotid media thickness, TG, TC, LDL-C, DD, PC, and hs-CRP were significantly lower (*P* < 0.05). The clinical effect of the study group was outstanding (*P* < 0.05). The defect rate of the study group was lower than that of the control group, but there was no difference (*P* < 0.05).

**Conclusion:**

Ezetimibe combined with medium- and low-intensity atorvastatin with aspirin in the treatment of cerebrovascular diseases can effectively improve the coagulation function of patients, reduce the level of inflammatory factors in patients, and improve the level of blood lipids in patients, with high safety and worthy of clinical application.

## 1. Introduction

Cerebrovascular disease is a variety of diseases that occur in the brain, mostly in the elderly, and there are many different types, the most common of which is ischemic cerebrovascular disease. These patients often suffer from dizziness, headache, blurred vision, and, in severe cases, aphasia and hemiplegia [1, 2]. The disease is treated clinically by drugs and surgery and has a high incidence of morbidity, mortality, and recurrence, so it should be treated as soon as possible to avoid serious effects on the patient's health and daily life. Aspirin and atorvastatin are the main drugs used in the treatment of this disease, but some patients are intolerant to these drugs, and the treatment is not satisfactory [3].

Ezetimibe is a cholesterol absorption inhibitor and is a similar lipid-regulating drug to atorvastatin, with selective inhibition of cholesterol absorption and anti-inflammatory effects [4]. Ezetimibe combines lipid-lowering agents: rosuvastatin, an HMG-CoA reductase inhibitor that has particularly strong inhibitory effects on hepatic cholesterol synthesis, and ezetimibe. Climent et al. [5] showed that ezetimibe combined with low- to medium-strength atorvastatin and aspirin treatment for cerebrovascular disease could improve the level of coagulation indexes and reduce the level of lipid indexes in patients, effectively improving their coagulation function and lipid metabolism, and with better safety of administration.

Therefore, in order to analyze the therapeutic effect of ezetimibe combined with low- to medium-strength atorvastatin and aspirin on cerebrovascular disease, 110 patients with cerebrovascular disease treated in our hospital from June 2020 to June 2021 were selected and reported as follows.

## 2. Materials and Methods

### 2.1. Study Subjects

110 patients with cerebrovascular disease treated in our hospital from June 2020 to June 2021 were selected and divided into 55 cases in the control group and 55 cases in the study group according to the lottery method, 25 males and 20 females in the control group, aged 42-74 years, mean age (57.45 ± 2.55), duration of disease (1-7 years), and mean duration of disease (4.23 ± 1.11 years). There were 28 males and 17 females in the study group, aged 43-78 years, mean age (58.56 ± 2.76), duration of disease 1-8 years, and mean duration of disease (4.66 ± 1.65 years), and the general data of the two groups were balanced and comparable (*P* > 0.05). All gave informed consent to the study, signed the informed consent form, and were approved by the ethics committee of our hospital.

### 2.2. Inclusion Criteria

(i) All were diagnosed with cerebrovascular disease by clinical imaging; (ii) all were aged ≥ 40 years.

### 2.3. Exclusion Criteria

The participant has (i) history of allergy or contraindication to the drugs to be used in this study, (ii) more serious cardiovascular disease and coagulation disorders, (iii) or other serious primary diseases.

### 2.4. Treatment of Patients

After a thorough examination, patients in the 2 groups should be given aspirin, size: 0.1 g × 7 tablets × 2 plates/box, oral medical treatment, dose: 100 mg/d. The control group should be treated with regular dose of atorvastatin on top of the above treatment, taken orally at bedtime, dose: 40 mg/d. The study group was treated with atorvastatin at a low to moderate dose of 20 mg/d orally at bedtime in addition to aspirin and with ezetimibe at 10 mg/d. Both groups were treated for 2 weeks.

### 2.5. Indicator Observation

(i) The ADL scale [6] was used to evaluate the patient's ability to perform activities of daily living (ADL): its score ranges from 14 to 56, with higher scores indicating higher ability to perform activities of daily living. (ii) The carotid artery intima-media thickness was measured and compared between the 2 groups of patients. (iii) Lipid level testing is as follows: the venous blood was taken from patients before and early morning after treatment, and lipid levels were measured using the rate method. (iv) Coagulation levels are as follows: DD, ATIII, and PC levels were measured using a fully automated biochemical analyzer, and hs-CRP levels were measured using an enzyme-linked immunosorbent assay. (v) Clinical effect is as follows: evaluation according to the condition of the patient: significant effect: significant improvement of clinical symptoms and normal indicators; effective: basic normal clinical indicators and improvement of indicators; ineffective: no improvement of clinical indicators, no change of indicators and serious condition. Effective rate = (effective + effective)/total number of cases × 100%. (vii) The adverse rates of the 2 groups were counted and compared.

### 2.6. Statistical Analysis

The SPSS22.0 statistical software was used to analyze and process the data. The measurement data were described by mean ± standard deviation ($\overset{-}{x}\pm s$), *t*-test for independent samples was used for comparison between groups, and repeated measures ANOVA was used for comparison before and after treatment. The count data were expressed as frequencies and percentages, the *χ*^2^ test was used for comparison between groups, and *P* < 0.05 was regarded as statistically significant difference.

## 3. Results

### 3.1. Comparison of ADL Scores and Carotid Artery Intima-Media Thickness between the 2 Groups

As shown in Table 1, there was no difference in cognitive function, ability to perform activities of daily living, and carotid artery intima-media thickness between the 2 groups before treatment (*P* > 0.05). After treatment and ADL scores increased and carotid artery intima-media thickness decreased (*P* < 0.05), and after treatment, ADL scores were higher, and carotid artery intima-media thickness was lower in the study group (*P* < 0.05).

### 3.2. Comparison of Blood Lipid Levels before and after Treatment in the 2 Groups

As shown in Table 2, there was no difference between the blood lipid levels of the 2 groups before treatment (*P* > 0.05). After treatment, TG, TC, and LDL-C levels decreased, and HDL-C levels increased (*P* < 0.05). The levels of TG in the control group were 4.21 ± 1.33 after treatment, while they were 2.04 ± 0.88 in the study group (*P* = 0.001). The levels of TC in the control group were 6.23 ± 1.24 after treatment, while they were 3.43 ± 0.55 in the study group (*P* = 0.001). The levels of LDL-C in the control group were 3.22 ± 0.55 after treatment, significantly higher than that in the study group (1.58 ± 0.53, *P* = 0.001).

### 3.3. Comparison of Coagulation Levels between the 2 Groups of Patients

As shown in Table 3, there was no difference in coagulation levels between the 2 groups of patients before treatment (*P* > 0.05); after treatment, DD, PC, and hs-CRP levels decreased, and ATIII levels increased (*P* < 0.05), and after treatment, DD, PC, and hs-CRP levels were lower, and ATIII levels were higher (*P* < 0.05).

### 3.4. Comparison of Clinical Outcomes between the 2 Groups of Patients

As shown in Table 4, the clinical outcome of the study group was outstanding. There are total 55 cases in the control group and the study group. There are 23 cases that are significant in the control group and 29 in the study group. The effective case in the control group was 17 and 23 in the study group. However, the invalid case in the control group was 15 and 3 in the study group. Therefore, the total efficiency in the study group is significantly greater than the control group (*P* = 0.002).

### 3.5. Comparison of Adverse Rates between the 2 Groups of Patients

As shown in Table 5, the study group had a lower adverse rate than the control group (*P* < 0.05). There are total 55 cases in the control group and the study group. There are 2 cases of nausea and vomiting in the control group and 1 in the study group. The poor appetite in the control group was the same as the study group. The muscle pain in the control group was 1, and none in the study group. Therefore, the total adverse reaction rates in the study group are significant lower than the control group (*P* = 0.0418).

## 4. Discussion

Cerebrovascular disease is mainly associated with hyperlipidemia, dense blood, and atherosclerosis, with capillary morbidity being more related to atherosclerosis. As a result of inflammation caused by atherosclerosis in the arteries, the endothelium of the patient's blood vessels is damaged, which in turn leads to poor lipid transport and large deposits that impede the flow of blood, subsequently causing hypoxia in the brain. The lack of oxygen in the brain directly affects the neurological function of the patient. Clinical medication is mostly used to control inflammation and inhibit platelet aggregation to improve the patient's symptoms and prognosis [7, 8].

This study showed that the ADL scores were higher and carotid intima-media thickness was lower in the study group after treatment. This result indicates that ezetimibe combined with low- to medium-strength atorvastatin supplemented with aspirin can greatly improve the cognitive function and quality of life of the patients. The results of a study by Sun et al. [9] showed that ezetimibe combined with rosuvastatin was clinically effective in treating early-onset coronary artery disease, effectively reducing serum MCP-1 and MIP-1*α* expression, regulating blood lipids, and improving cardiac function without increasing adverse effects. In this paper, TG, TC, and LDL-C levels were lower, and HDL-C levels were higher in the study group after treatment. TG, TC, LDL-C, and HDL-C are all lipid indicators that reflect the patient's lipid metabolism. Atorvastatin can effectively inhibit cholesterol synthesis and reduce the myocardial damage caused by LDL and treacherous cholesterol in serum, exerting its lipid-regulating effect, but high doses alone can significantly reduce LDL-C levels in patients and increase the risk of adverse effects [10, 11]. Ezetimibe binds to and inhibits the activity of NPCILI in humans, thus blocking intestinal absorption of cholesterol and, in combination with atorvastatin, can have a better effect on regulating lipid levels. Ogiso et al. [12] showed that ezetimibe combined with pitavastatin for the treatment of coronary heart disease could effectively improve the efficacy, improve lipids and carotid plaque, reduce hs-CRP and CX3CR-1 expression, and improve endothelial cell function in patients, resulting in clinical benefits for patients with coronary heart pain, consistent with the findings of this paper.

In this paper, the low levels of DD, PC, and hs-CRP and the high levels of ATIII after treatment were analyzed because DD is a degradation product that reflects whether the body is in a hypercoagulable state and secondary hyperfibrinolytic state. ATIII is a natural anticoagulant protein with consistent thrombin activity [13]. PC has a platelet clotting effect, and hs-CRP is part of the body's nonspecific mechanism, which can better reflect the presence of inflammatory state of the body. Aspirin can effectively reduce platelet aggregation and inhibit thrombus formation [14]. Atorvastatin is a reductase kinase, which can reduce hypercholesterolemia and impaired lipid metabolism by inhibiting the synthesis of hydroxymethylglutaryl coenzyme A. It normalizes vascular metabolism in patients, reduces damage to the vascular endothelium, and decreases the inflammatory response [15]. While the effect of different doses of atorvastatin varies, treatment with high-intensity atorvastatin alone with aspirin may cause more adverse effects to patients [16, 17]. Ezetimibe is a cholesterol inhibitor, which can eliminate cholesterol in the blood in a timely manner and play an anti-inflammatory and endothelial protective role. The combination of this drug with regular doses of atorvastatin and aspirin treatment can greatly reduce the adverse effects caused by atorvastatin and enhance the protection of endothelial vessels, so that patients do not have platelet aggregation and reduce the inflammatory response of patients [18–20].

The advantage of this study is to show that the adverse rate in the study group was lower than that in the control group. This result indicates that ezetimibe combined with low- to medium-strength atorvastatin adjuvant to aspirin has a better safety profile in cerebrovascular disease and is worthy of clinical promotion. However, there are also limits. First, the number of patients is not enough. Second, the mechanism is not clarified in this study. Further researches are needed to study more.

## 5. Conclusion

In conclusion, ezetimibe combined with low- to medium-strength atorvastatin and aspirin is effective in improving the coagulation function, reducing the level of inflammatory factors, and improving the lipid level of patients in the treatment of cerebrovascular disease, with high safety and worthy of clinical promotion.

## Figures and Tables

**Table 1:** Comparison of ADL scores and carotid artery intima-media thickness between the 2 groups ($\overset{-}{x}\pm s$).

Group	Cases (*n*)	ADL score (points)		Carotid artery intima-media thickness	
		Pretreatment	Posttreatment	Pretreatment	Posttreatment
Control group	55	44.28 ± 7.03	58.78 ± 8.32	1.53 ± 0.45	1.33 ± 0.21
Study group	55	44.21 ± 7.66	69.20 ± 9.89	1.56 ± 0.67	1.11 ± 0.21
*t*		0.050	5.979	0.276	5.494
*P*		0.960	0.001^∗^	0.783	0.001^∗^

**Table 2:** Comparison of lipid levels before and after treatment in the 2 groups (($\overset{-}{x}\pm s$), mmol/L).

Group	Cases (*n*)	TG		TC		HDL-C		LDL-C	
		Pretreatment	Posttreatment	Pretreatment	Posttreatment	Pretreatment	Posttreatment	Pretreatment	Posttreatment
Control group	55	5.23 ± 2.11	4.21 ± 1.33	7.27 ± 2.11	6.23 ± 1.24	2.13 ± 0.77	2.11 ± 0.78	5.23 ± 1.44	3.22 ± 0.55
Study group	55	5.12 ± 2.43	2.04 ± 0.88	7.15 ± 1.67	3.43 ± 0.55	2.22 ± 0.56	3.02 ± 0.21	5.32 ± 1.01	1.58 ± 0.53
*t*		0.254	10.090	0.331	15.310	0.701	8.355	0.380	15.920
*P*		0.800	0.001^∗^	0.741	0.001^∗^	0.485	0.001^∗^	0.705	0.001^∗^

**Table 3:** Comparison of coagulation levels between the 2 groups ($\overset{-}{x}\pm s$).

Group	Cases (*n*)	DD (mg/L)		ATIII (%)		PC (mg/L)		hs-CRP (mg/L)	
		Pretreatment	Posttreatment	Pretreatment	Posttreatment	Pretreatment	Posttreatment	Pretreatment	Posttreatment
Control group	55	2.62 ± 0.34	0.77 ± 0.25	72.13 ± 11.23	82.21 ± 7.34	23.14 ± 4.01	14.36 ± 3.36	7.88 ± 1.65	4.77 ± 1.35
Study group	55	2.65 ± 0.55	0.33 ± 0.04	73.12 ± 11.11	97.45 ± 7.33	21.12 ± 4.08	8.78 ± 3.09	7.16 ± 1.37	3.03 ± 0.21
*t*		0.344	12.890	0.465	10.900	2.619	9.065	2.490	9.445
*P*		0.731	0.001^∗^	0.643	0.001^∗^	0.010^∗^	0.001^∗^	0.014^∗^	0.001^∗^

**Table 4:** Comparison of clinical outcomes between the 2 groups of patients (cases, %).

Group	Cases (*n*)	Significant effective	Effective	Invalid	Total efficiency
Control group	55	23	17	15	40 (72.72)
Study group	55	29	23	3	52(94.54)
*χ* ^2^					9.565
*P*					0.002^∗^

**Table 5:** Comparison of adverse rates as well as recurrence rates in the 2 groups (cases, %).

Group	Cases (*n*)	Nausea and vomiting	Poor appetite	Muscle pain	Adverse reaction rates
Control group	55	2	1	2	5 (9.09)
Study group	55	1	1	0	2 (3.63)
*χ* ^2^					1.373
*P*					0.241

## Data Availability

The data used to support this study are available from the corresponding author upon request.
